# Machine Learning Technology-Based Heart Disease Detection Models

**DOI:** 10.1155/2022/7351061

**Published:** 2022-02-27

**Authors:** Umarani Nagavelli, Debabrata Samanta, Partha Chakraborty

**Affiliations:** ^1^Dayananda Sagar Research Foundation, University of Mysore (UoM), Mysore, Karnataka, India; ^2^Department of Computer Science, CHRIST (Deemed to be) University, Bangalore, Karnataka, India; ^3^Department of Computer Science and Engineering, Comilla University, Cumilla-3506, Bangladesh

## Abstract

At present, a multifaceted clinical disease known as heart failure disease can affect a greater number of people in the world. In the early stages, to evaluate and diagnose the disease of heart failure, cardiac centers and hospitals are heavily based on ECG. The ECG can be considered as a regular tool. Heart disease early detection is a critical concern in healthcare services (HCS). This paper presents the different machine learning technologies based on heart disease detection brief analysis. Firstly, Naïve Bayes with a weighted approach is used for predicting heart disease. The second one, according to the features of frequency domain, time domain, and information theory, is automatic and analyze ischemic heart disease localization/detection. Two classifiers such as support vector machine (SVM) with XGBoost with the best performance are selected for the classification in this method. The third one is the heart failure automatic identification method by using an improved SVM based on the duality optimization scheme also analyzed. Finally, for a clinical decision support system (CDSS), an effective heart disease prediction model (HDPM) is used, which includes density-based spatial clustering of applications with noise (DBSCAN) for outlier detection and elimination, a hybrid synthetic minority over-sampling technique-edited nearest neighbor (SMOTE-ENN) for balancing the training data distribution, and XGBoost for heart disease prediction. Machine learning can be applied in the medical industry for disease diagnosis, detection, and prediction. The major purpose of this paper is to give clinicians a tool to help them diagnose heart problems early on. As a result, it will be easier to treat patients effectively and avoid serious repercussions. This study uses XGBoost to test alternative decision tree classification algorithms in the hopes of improving the accuracy of heart disease diagnosis. In terms of precision, accuracy, f1-measure, and recall as performance parameters above mentioned, four types of machine learning (ML) models are compared.

## 1. Introduction

Cardiovascular disease (CVD) is a type of heart disease that continues to be a major cause of death worldwide, accounting for over 30% of all deaths. If nothing is done, the total number of fatalities in the world is anticipated to rise to 22 million by 2030. Plaques on arterial walls can obstruct blood flow, resulting in a heart attack or stroke. Heart disease is caused due to various risk factors such as physical inactivity, unhealthy diet, and the effective use of alcohol and tobacco [1, 2]. The abovementioned factors are reduced by adopting a good daily lifestyle, namely, reducing salt in the diet, consumption of vegetables and fruits, practicing physical activity regularly, and discontinuing alcohol and tobacco use, which helps to minimize the risk of heart disease [3]. The solution to overcome these problems is to use the collection of patient records from different health care centers and hospitals. For getting the results and seeking another opinion from an experienced doctor the decision support system is used. The unnecessary test conductions are avoided by this technique for diagnosis, thereby saving money and time [4, 5]. Recently, a system of hospital management was utilized for managing the health care or patient data which means more data are produced by these systems. For predicting heart disease, the DSS utilizing the NB (Naïve Bayes) algorithm was developed. A web application is constructed to obtain the application and user input, and it retrieves key features relating to heart disease from a historical database (the Cleveland data set) [6, 7].

More number of neurohormonal regulatory mechanisms are triggered in the initial stages of heart failure disease (HFD). In a short duration, these compensatory mechanisms can cause the HFD consequences, leading to accentuated ventricular dysfunction, dyspnea on exertion, peripheral edema, pulmonary, and heart remodeling which can cause afterload and preload permanent changes. More options of treatment with HFD are given to the patient including lifestyle changes and implantable or medication devices such as a defibrillator or pacemaker. The main concern is ensuring the follow-up in this population given that hospitalization due to acute HFD decompensation is the leading cause of healthcare expenditure. Statistics and studies show that heart diseases are the most significant issue faced by people particularly HFD [8, 9]. For various diseases, early diagnosis and detection of cardiac disease is the first step in care and treatment.

The HFD is now an emerging disorder for diseases such as hypertension, insomnia, and heart disease among others. The HFD detection on ECG is completed through variations detection in duration of heart beats from the time interval from 1 wave of PQRST to the next wave of PQRST. For IHD early detection, an emerging and promising noninvasive diagnostic tool is MCG (Magenetocardiography). While MCG is less influenced by contact interference of electrode-skin compared to ECG, it is highly sensitive to vortex current and tangential causes through the tissue of ischemic cardiac. Despite its high signal quality, MCG interpretation is time-consuming, highly dependent on interpreting experience, and has limited appeal in clinics. As a result, clinicians would benefit from an autonomous system that can detect and localize ischemia at an early stage [10].

Early identification of heart disease of improved diagnosis and high-risk individuals using a prediction model can be recommended generally for fatality rate reduction, and decision-making is improved for further treatment and prevention. In CDSS, a prediction model is implemented and utilized to support the clinicians in assessing the heart disease risk, and appropriate treatments are provided for managing the further risk. Additionally, numerous studies have also reported that CDSS implementation can improve decision quality, clinical decision making, and preventive care, respectively [9, 11]. Coronary artery disease (CAD), also known as ischemia heart disease (IHD), is the leading cause of death in adults over the age of 35 in different countries. During the same time span, it became China's biggest cause of death. When blood flow to the heart is reduced due to coronary artery stenosis, IHD occurs. Myocardial damage can have serious consequences including ventricular arrhythmia or even sudden cardiac death due to myocardial infarction.

### 1.1. Major Contribution of Research

Machine learning may be used to diagnose, detect, and forecast many disorders in the medical industry. The primary purpose of this study is to give clinicians a tool to detect cardiac problems at an early stage. As a result, it will be easier to deliver appropriate treatment to patients while avoiding serious effects. This study uses XGBoost to test several decision tree classification algorithms in the hopes of improving performance in heart disease diagnosis.

The remaining paper is organized as follows: In Section 2, literature analysis is presented. ML techniques for heart disease prediction is presented in Section 3. Feature extraction is projected in Section 4. Heart disease prediction using the XGBoost algorithm is elaborated in Section 5. Results are shown in Section 6. The concluding remarks are given in Section 7.

## 2. Literature Analysis

In the system of the human heart, the heart's electrical activity is recorded by ECG with various wave forms through skin electrodes. For heart disease identification, it is a noninvasive technique which reflects heartbeat, heart rate, and cardiac health. The number of cells in the human body has no direct contact with the outer location. Moreover, they depend on the cardiovascular system for serving as a provision of transport for them. In system of cardiovascular, the fluids are two kinds are flow through it. Blood is the first fluid type. Here, the circulatory system forms the blood vessels and heart. Lymph is the second type of fluid. The structure of the lymphatic system is formed by lymph nodes and lymphatic vessels. The cardiovascular system can be formed by the combination of the lymphatic system and the vascular system [12]. In heartbeat, a heart cycle is an action series. A heart cycle typically contains both atria, with each ventricle contraction synchronized a fraction of a second later. The heart is produced and interconnected using heart muscle cells, so when one of them contracts, it causes nearby cells to excite. The muscles rest between beats in the cardiac cycle, which contributes to aerobic breathing. Two parts are there, which are further discussed in this study.

### 2.1. Part 1 Is ‘Systole'

It is the expression for contraction. It happens whenever the ventricles are in the stage of contracting and cause the blood to pump into the vessels of the heart with A–V valves closure and semilunar valves opening.

### 2.2. Part 2 Is ‘Diastole'

It is an expression for relaxation. It happens whenever the ventricles are in a stage of relaxing. This causes back-blood pressure to the valves of the closing semilunar and opening valves of A–V, respectively.

Previous studies have shown promising results for CVD automatic detection. But still, there are a few concerning problems. Firstly, studies utilizing private datasets suffer from variations of database and small-sized databases, especially for MCG studies in which larger public datasets are unavailable. However, based on public datasets, ECG studies might not accomplish equal performance if they are transferred from benchmark to clinical domain. Representatives composes the public datasets of ECG. The ECG datasets easily identify abnormal cases and would be biased to perform early diagnosis [13]. On model performance, feature selection has shown a significant impact. Past studies presented features from three categories: (a) information theory features, (b) time domain features, and (c) frequency domain features.

Every category is represented as effective and has the ability for revealing some complicated aspects of cardiac electrophysiological signals. Certain studies are carried out to evaluate the significance of different features. For solving this issue a large feature group is relatively designed that contains abovementioned two categories. Through the feature importance weight analysis, the following is determined:

- Repolarization synchronicity of T wave is described by features as a core feature for identifying the subjects of IHD
- Features describe that the characteristics of the magnetic pole are associated with coronary stenosis locations

Various studies are reporting that the heart disease diagnosis development based on models of ML can provide the objective of HDPM with improved performance. The 2 publicly available datasets of heart disease such as Cleveland and Statlog are mostly used for comparing the prediction models' performance between researchers. In the area of healthcare, ML-based clinical decision making has been applied recently. In machine learning, recent advances are representing discriminative classifiers' advantages for cardiac disease automatic detection. Studies have previously shown that machine learning algorithms, namely, SVM, RF (random forest), LR (logistic regression), BPNN (back propagation neural network), and MLP (multilayer perceptron) are utilized successfully for decision-making tools to predict heart disease based on individual information. Various studies revealed the hybrid model merits that achieved good performance in heart disease prediction, namely, RF with a linear model, MLP, Bayes Net (BN), majority voting of NB, and RF and two stacked SVMs, respectively [14]. Kalia Orphanou et al., in the NB classification model, the TARs (Temporal Association Rules) feature is used for diagnosing heart disease. To preprocess the data, a temporal abstraction (TA) is used and a temporal pattern mining algorithm is utilized for finding TARs by frequent temporal relationships identification between TAs. In Naïve Bayes classifier, periodic TARs are considered as features finally. With the help of possible recurrence of each TAR pattern with relevant patient history, an 82% accuracy is obtained. Theresa Princy et al. have conducted a survey on several machine learning techniques which are utilized to predict the heart diseases risk of a person depending on various attributes such as gender, age, cholesterol, and pulse rate. When increasing the accuracy of risk and attributes, the author can use the analysis of the K-nearest neighbour algorithm, Naïve Bayes, and neural network. The accuracy is increased with a low number of attributes, which is possible by using various methods [15]. Prerana et al. predicted the risk level of probabilistic analysis and classification (PAC) and heart disease completed by machine learning technique. For handling patients' records and various machine learning algorithms analysis, the map reduce programming is used and given with the graphical representation. In the cloud, this approach is available and globally accessible. Furthermore, it can be extended for determining different diseases such as cancer, diabetes, brain tumor, and so on. Shadab et al. use the technique of NB data mining for supporting the users to know the answers for predefined questions in the application of web based. For diagnosing heart disease, doctors use these intelligent decisions when NB algorithm accuracy can be improved by utilizing various techniques [16].  Figure 1 shows ML techniques for heart disease prediction.

## 3. ML Techniques for Heart Disease Prediction

### 3.1. Naïve Bayes Weighted Approach (NBwa)

The web application is the proposed system. It can be classified into two modules: admin side and user side, respectively. The admin submitted the dataset into the database in the form of an excel sheet, which was then translated into weights and stored. Clusters were formed from the records. Depending on average weight or each of the clusters is determined, attribute (vessel) classification and in the database this feature can be stored. Using provided fields, the user inputs and patient data are converted into weights, and the algorithm of NB is applied to the data. The result can be displayed to the user based on system probability. Various events' conditional and marginal probabilities are compared by the Naïve Bayes algorithm. For the given samples, this algorithm is useful for calculating the possible nearest value [17]. The Bayes theorem is useful for calculating the diagnostic probability when the patient's health is monitored based on a few symptoms. The Bayes rule is used in a variety of data mining approaches. This technique is more beneficial for developing predictive capability models and provides a variety of ways to examine and explore the data. The Naïve Bayes classifier is an appropriate scheme when a given input attribute is more. Compared to many other classification techniques this algorithm is simple, but it has better performance. The heart disease patient's characteristics are easily identified by the Naïve Bayes classifier technique. This algorithm will find the input attributes' probability during a predictable disease state [18].  Figure 2 shows ML techniques for heart disease prediction.

### 3.2. Magnetocardiography-Based Ischemic Heart Disease Detection

The framework of ischemic heart disease detection using ML classifiers is shown in Figure 3. The feature groups show that Pearson's coefficient was used to create a heatmap to investigate the association between characteristics and the target variable. Similar data points were grouped to evaluate clustering strength in order to investigate the links exhibited in the heatmap. With a mapping of the target variable, age and systolic blood pressure were grouped. This makes it easier to see the target variable's distribution. Preprocess the raw MCG signals for T-wave segmentation, filtering, and averaging [19, 20]. Then, 3 feature categories are extracted. Few of these features would be redundant, but still they are included in the classification procedure because past studies suggest that ML algorithms like SVM are not sensitive to redundant features' presence. On the other hand, omitting significant features is more hazardous than nonimportant features.

## 4. Feature Extraction

### 4.1. Time Domain

Time domain 18 features are summarized for describing the following:

1. Maximum cardiac current characteristics
2. Pattern of magnetic field map
3. Distribution of negative/positive magnetic poles in the TT interval is independently distributed with a normal distribution that has a mean of 0 and constant variance

In addition, 6 related features of magnetic poles are presented to describe the following: change of negative/positive pole area in T wave and displacement of negative/positive in T wave. In the following study, it was determined that they were associated with the location of stenosis. Interesting characteristics of features from 2 aspects: dynamic changes and values at the peak of the T-wave during the interval TT. For achieving this, the interval TT is partitioned into 24 shorter subwindows, from which 18 time features are extracted.

### 4.2. Discrete Wavelet Transform Domain

A db-4 (Daubechies 4) DWT is applied with 4 levels on each of the 36 channels. The signal is decomposed into time-frequency components through DWT. The 4^th^ level DWT low frequency part (A4 component, corresponding from 0 to 7.8 Hz approximately) is reconstructed utilizing IDWT (inverse DWT).

### 4.3. Information Theory

Based on the theory of electrophysiology, ischemic subjects' signal perturbation during the segment ST is higher than that of healthy persons. The 3 measures are selected from the following: (i) for each channel Shannon entropy, (ii) multidimensional Gini index, and (iii) entropy of SVD (singular value decomposition).

## 5. Heart Disease Prediction Using the XGBoost Algorithm

Develop HDPM for providing high prediction performance, absence/presence of heart disease, and to provide the present situation of a patient. The development process of HDPM is represented through flow chart which is shown in Figure 4. Firstly, collect the datasets of heart disease. Secondly, data preprocessing is carried out for the transformation of data. Third, apply the outlier detection based DBSCAN technique for determining the outlier data provided by optimal parameters [21]. Fourth, from the training dataset, remove the detected outlier data. Fifth, for balancing the training dataset, utilize SMOTE-ENN based data balancing technique. Sixth, to learn from the training dataset and for generating HDPM using MLA based on XGBoost. The main parameter with adjustment with max_depth_ = 5, min_childweight_ = 1, gamma = 0, subsample, colsample_bytree_ = 0.8, and scale_posweight_ = 1. Finally, for evaluating the presented model performance, performance metrics are presented. Within the CDSS, HDPM is generated [22, 23]. In this study, a 10-fold cross-validation technique is utilized for avoiding overfitting. The models are allowed by cross-validation to learn from various training datasets through repeated sampling. Therefore, data maximizing is utilized for validation, which helps for overfitting prevention. Past studies have demonstrated that the 10-cross field validation technique will be utilized for maintaining the bias variance trade-off that eventually provides a generalized model and protects against overfitting [24]. The proposed heart disease prediction model using XGBoost is shown in Figure 4.

## 6. Results

Different machine learning methods use different datasets with independent specification. Total 50 test cases are used in the prediction of heart diseases in the paper. Among these 50 test cases, 6 are false negatives, 1 is false positive, 18 are TPs, and 25 are TNs [25]. The collection of data is part of cardiovascular disease retrospective studies utilizing the recordings of multichannel MCG. There are 227 people with coronary stenosis and 347 people who are healthy in the database. There are 16 NSTEMI (non-ST-elevation myocardial infarction) instances in the sample. For the ischemic group, coronary angiography is performed. There were 227 IHD patients (left anterior descending) [26].

Several datasets are used to demonstrate the presented approach's capacity to detect HFD using ECG signals. The proposed method is tested on 38 real data recordings of ECG signals with HFD from the PhysioNet database. Consider the 5-section (P, *Q*, R, S, and T) segmentation issues of the ECG signal for each round [27]. It is also regarded as the three distinct zones (QRS, *T*, and P) that provide varying probabilities of peak-peak and all-waves time interval borderlines in the patient's ECG [21, 28, 29]. It has been discovered that three components of the processed ECG signal are segregated and distributed in the same way. For every patient with HFD, the ISVM-DO will identify all P, *Q*, R, S, and *T* wave peak values in the ECG waveform. As a result, the system extracts essential morphological aspects from processed ECG. Many random tests and cross-validation tests are used to train the proposed method predictor on 125 samples from the training dataset [30, 31].

For exploring how heart illness is recognized using an ML approach, two datasets of heart diseases (Cleveland and Statlog; termed datasets I and II) are used. Although the original dataset comprises 79 raw attributes and 303 subjects, only 13 of them are utilized, and just one attribute is used as an output class. The remaining 297 subjects are used in the preprocessing step after 6 subjects were excluded from the dataset due to missing values. The XGBoost V0.81 Python library is used to implement XGBoost. Using the DBSCAN technique, remove outlier data from heart disease training datasets. The software XGBoost is used to generate HDPM [2, 32]. To evaluate the performance of ML techniques, 4 different parameters are utilized: recall, F1-measure, accuracy, and precision. For measuring the potential of these 4 parameters a confusion matrix is utilized from the model: *F*_*n*_ (false negative), *T*_*n*_ (true negative), *F*_*p*_ (false negative), and *T*_*p*_ (true positive). Number of subjects classified correctly as “positive” (heart disease presence) is known as *T*_*p*_, number of subjects classified correctly as “negative” (absence/healthy heart disease) is represented as *T*_*n*_. Similarly, number of subjects classified incorrectly as “negative” (when they have heart disease) is represented as *F*_*n*_, and number of subjects classified incorrectly as “positive” when they not having heart disease is represented as *F*_*p*_.

### 6.1. Accuracy

The ratio of accurately predicted predictions by the model to all types of completed predictions in the problem classification is known as accuracy.

(1) $$\begin{array}{c} \text{Accuracy}=\frac{\left(T_{p}+T_{n}\right)}{\left(T_{p}+T_{n}+F_{p}+F_{n}\right)}. \end{array}$$

### 6.2. Precision

Precision or positive predictive is defined as the ratio of accurate positive scores (*T*_*p*_) to the total number of positive scores (*T*_*p*_ + *F*_*p*_) predicted by the classification algorithm.

(2) $$\begin{array}{c} \text{Precision}=\frac{T_{p}}{\left(T_{p}+F_{p}\right)}. \end{array}$$

### 6.3. Recall

The recall can be defined as the ratio of accurate *T*_*p*_ to the total *T*_*p*_ “+” *F*_*n*_.

(3) $$\begin{array}{c} \text{Recall}=\frac{T_{p}}{\left(T_{p}+F_{n}\right)}. \end{array}$$

### 6.4. F1-Measure

The F1-measure is a function of precision and recall. F1 must be 1 for the classification algorithm's good performance and 0 for bad performance.

(4) $$\begin{array}{c} \text{F}1-\text{measure}=2\times \frac{\left(\text{precision}*\text{recall}\right)}{\left(\text{precision}+\text{recall}\right)}. \end{array}$$

Different ML techniques-based heart disease detection performance is evaluated with the different parameters, and these values are shown in Table 1.

The graphical representation of different ML techniques to predict heart disease in terms of accuracy and precision parameters is represented in Figure 5.

The graphical representation of the different ML techniques to predict heart disease in terms of recall and F1-measure parameters is represented in Figure 6.

From the abovementioned table and graphs, it is clear that the accuracy parameter is high in the XGBoost algorithm-based heart disease detection and low in the Naïve Bayes with weighted approach.  Table 2 shows confusion metrics analysis for applying classifier.

## 7. Conclusion with Future Work

The survey on machine learning technology-based heart disease detection models is provided in this paper. Four approaches of ML models for heart disease detection are analyzed in this survey; these are the Naïve Bayes with weighted approach based prediction, 2 SVM's with XGBoost based prediction, an improved SVM (ISVM) based on duality optimization (DO) technique based prediction, and an XGBoost based prediction. According to the results analysis, the accuracy, precision, recall, and F1-measure parameters are high in the XGBoost algorithm-based heart disease detection and only accuracy is low for the Naïve Bayes with weighted approach than others, and the remaining precision, recall, and F1-measure values are low in SVM with duality optimization (DO) model. The present survey paper gives the best idea regarding different machine learning-based heart disease detection methods.This research can be updated in the future by adding more attributes to the heart disease dataset and making it more interactive for the users. It can also be carried out as a mobile application with reduced computing time and complexity. We will make changes to the system by linking it to the hospital's database.

## Figures and Tables

**Figure 1:** System architecture.

**Figure 2:** ML techniques for heart disease prediction.

**Figure 3:** Framework of ischemic heart disease detection.

**Figure 4:** Proposed heart disease prediction model using XGBoost.

**Figure 5:** Different ML methods in terms of accuracy and precision.

**Figure 6:** Different ML methods in terms of recall and F1-measure.

**Table 1:** Comparative analysis of different machine learning methods.

Methods	Accuracy	Precision	Recall	F1-measure

Naïve Bayes weighted approach	86.00	82.34	87.25	89.21
2 SVM's and XGBoost	94.03	86.56	94.78	92.79
SVM and DO	89.4	66.1	81.3	82.1
XGBoost	95.9	97.1	94.67	95.35

**Table 2:** Confusion metrics analysis for applying classifier.

Model name	Label	Predictive negative	Predictive positive

Naïve Bayes and weighted approach	Actual negative	6314	6214
	Actual positive	5076	5142

2 SVM's and XGBoost	Actual negative	6314	6014
	Actual positive	5410	5142

SVM and DO	Actual negative	5897	5001
	Actual positive	4517	4221

XGBoost	Actual negative	5794	5001
	Actual positive	4876	4221

## Data Availability

The heart disease data that support the findings of this study are available on request from the corresponding author.
